This article has been retracted.

# Application and Analysis of Big Data Mining in the Foreign Affairs Translation System

**DOI:** 10.1155/2022/8216522

**Published:** 2022-11-19

**Authors:** Chaowei Zhang

**Affiliations:** School of English and International Studies, Beijing Foreign Studies University, Haidian, Beijing 100089, China

## Abstract

Based on the expansion of scientific and technological capabilities, the trend of global integration has further strengthened, and the relations between countries have become closer and closer. Therefore, the foreign affairs translation system plays a very important role. Many scientific and technological projects have carried out research and analysis around the foreign affairs translation system. Nowadays, the wide variety of data and the complexity of languages in various countries force the processing structure of the foreign affairs translation system to be changed to adapt to the development of big data. In this context, this article studies the foreign affairs translation system based on big data mining technology and designs the application of a new foreign affairs translation system model. The results of the experiment are as follows: (1) The development status of big data mining technology and the problems existing in the current foreign affairs translation system are analyzed, and the research direction of the experiment is determined. The foreign affairs translation system is analyzed according to big data mining technology, which determines the technical guarantee for the research of this article. (2) In keeping with the traditional effective foreign affairs translation system, this article uses big data mining algorithm analysis, the fuzzy c-means clustering algorithm, and the BP neural network algorithm to identify and analyze the problems of the foreign affairs translation model about data analysis ability technology, which quickly and accurately analyzes the problems of the system and optimizes and improves according to the specific problems.

## 1. Introduction

Viewing similar projects is very important to avoid duplication in project approval. However, there is no way to effectively find similar projects. A similarity detection method for scientific projects based on big data mining and multisource information integration is proposed. Using this method, the author studies a huge data network composed of project information, published papers, experts and institutions, and keywords. Multisource information should be integrated and a project similarity detection model should be established. Hadoop is used to accelerate data search. This article advances the model of project similarity detection and its key problems. It is hoped to provide new ideas and methods for finding similar projects in scientific project management [1]. A design method of the personalized recommendation system for the mobile game platform about data search is advanced. At the same time, the cosine similarity algorithm is used to enhance the game similarity. On this basis, a game model optimization method based on the combination of the genetic algorithm and K-means clustering is proposed to improve the defects of the traditional K-means algorithm, accelerate the convergence speed, and reduce the search space. Finally, the above conclusions are verified by experiments. This mechanism can effectively improve the accuracy of the game recommendation, increase user stickiness, and bring greater value to the game platform [2]. This article describes the relevant theoretical knowledge of big data and big data mining, and in view of the poor effect of data resources acquisition when university libraries provide services at present, through the technical support with the research goal of the collecting survey and connecting technical theory, this article simulates a library system model that provides personalized services. This article focuses on how to conduct a collective survey based on the user's behavioral characteristics and how to introduce the minimum feasibility to improve the premise of connecting the technical algorithm theory [3]. A new idea of tracking power grid faults on data analysis ability is proposed. It processes these discarded data by placing the damaged data into the variable area. This method can solve the problem of massive data processing. The combination of support vector machine and rough set theory is used to realize fault detection and diagnosis. When a faulty component is detected, the decision tree is used to guard or cut off the sensor fault if necessary. The cause of the fault should be analyzed and the function of the fault diagnosis system [4] should be optimized. Model exploration and big data learning are important technical methods for erosion exploration. The biggest difficulty in erosion learning research is how to effectively calculate the retention ability of erosion objects in the erosion environment. Erosion research should be combined with big data to investigate and analyze the erosion of complex data and calculate and infer the erosion process and erosion time. The combination of the two will be invested in the erosion change of special resources and the development of resource structure in the erosion environment. In this article, erosion and big data estimation methods were used to investigate the erosion of rare natural resources [5]. Based on the practical test and analysis of the educational achievements of logistics management, this article uses the situation analysis method to make a statistical investigation of the educational environment of logistics management and designs a set of the educational model of logistics management under the big data environment. The design of this model can not only help students majoring in logistics management to study their majors but also supplement and optimize according to the vacancies in the original education system, so as to improve the perfection and effectiveness of the education system [6]. The effective extension of urban diplomacy cannot be achieved without the efforts of the foreign affairs translation team. Foreign affairs translation is a complex and meticulous work, which requires translators to have rich professional knowledge and good foreign language ability. However, at present, there is a serious shortage of foreign interpreters in China; however, this cannot meet the demand of social construction for technical talents to a certain extent. All the time, foreign affairs translation operation has become increasingly administrative, which greatly restricts the cultivation of professional quality of foreign affairs translation, a special professional team. All-round innovative practice and scientific planning make the systematic project of foreign affairs translation team construction more and more perfect and organically adapt to the rapid development of urban diplomacy, which is an urgent task for local foreign affairs departments to study and solve [7]. With the development of social economy, there are more and more foreign affairs activities, the status of foreign affairs translation is becoming more and more important, and the demand for foreign affairs translation is becoming more and more urgent. At present, there are few foreign affairs translation papers in the system, and the foreign affairs translation papers that can be completed usually focus on one or two aspects. This article comprehensively and systematically expounds foreign affairs translation from the aspects of its definition, characteristics, standards, translation, and interpretation, as well as the qualification requirements of foreign affairs translators [8]. Today, with the internationalization of higher education development, it is increasingly obvious that higher education should have better foreign affairs communication ability. With the increasingly close relationship between China and the international community and the increasingly frequent foreign exchanges, higher requirements are put forward for the foreign language quality of talents, which also provides broad prospects and development space for colleges and universities to cultivate compound talents. Language structure, lexical meaning, emotion, and expression are important components of foreign affairs translation and the main obstacles to translation. Excellent translators should fully understand the cultural background of both sides, improve their knowledge and cultural level and comprehensive quality, and flexibly use their skills, so as to supply a good safeguard for the smooth growth of foreign affairs [9]. In the context of economic globalization, the internationalization of higher education is the general trend. The state encourages and supports institutions of higher learning to strengthen international exchanges and cooperation and further promotes international cooperation and learning between school educations. In the process of foreign exchange, due to different languages, oral expression of interpretation is grasped. This article summarizes the characteristics of foreign affairs interpretation and discusses the preparation before foreign affairs interpretation from the following two aspects: long-term translation preparation and short-term preparation [10]. Under the growth of social reform, the exchanges between local governments and foreign countries in all aspects are increasing, and the tasks of foreign affairs are also increasing year-by-year. In addition, the state has paid more attention to publicity and education; they should not only be proficient in foreign languages but also be competent for the important task of external publicity. We should understand both policies and business. Therefore, it is particularly important to do a good job of foreign affairs translation in colleges and universities. Some college teachers and other social translators are increasingly involved in foreign affairs translation. Therefore, it is particularly important to cultivate the quality of foreign affairs translators. Based on the standards of foreign affairs translators, this article emphasizes the quality requirements of foreign affairs translators and introduces the self-cultivation methods of foreign affairs translators. The improvement of political quality, professional quality, and comprehensive quality [11] should be emphasized. In oral translation, timeliness is the most significant one. To do a good job in interpretation, interpreters should not only have a high level of foreign language and skilled professional skills but also have strong adaptability and good psychological quality. Foreign affairs are high-quality translation. If foreign affairs translators want to be competent for this job, they must have solid basic knowledge of foreign languages and a lot of professional knowledge. Language is a communication tool, and the fundamental reason of language lies in the communication between people. Due to historical, ethnic differences, geographical environment, and other factors, all countries in the world, various national customs, have their own characteristics and language culture. Language is meaningless to each other. In the process of mutual communication, there is always no medium. Such a medium is to reduce but not increase the communication between the two sides. The medium without intention is translation [12]. The research shows that BIM technology can effectively improve the efficiency of railway construction and shorten the construction period; at the same time, it can also reduce the cost and waste of resources. Combined with specific engineering examples, the conclusion shows that this method is feasible and effective. It lays the foundation for the large-scale BIM platform of all stages of railway construction projects, including unified data standards and research and development, covering all stages and disciplines [13]. The functionalization of the synchronous inductor and asynchronous inductor is introduced, and these two inductors are put on the vertical elevator for practical testing. In addition, the configuration of the longitudinal inductor induction device is proposed and designed, which is an important part of the elevator model. As for the configuration of the inductor induction device, the experiment shows that its functionality is beyond doubt for the elevator. Through the comparative analysis of the synchronous sensor and asynchronous sensor, the shortcomings and optimization space between the two sensors are obtained [14]. Big data technology has a great impact on industry enterprises in today's era. Through a brief description of the concept and characteristics of big data analysis, the impact of big data on enterprises should be analyzed, the gaps in big data technology should be feed backed, specific problems should be solved, and finally the development trend of data analysis ability should be looked forward to. Starting from data analysis ability, this article studied the core content of data analysis ability-data mining technology and discusses the specific application methods of data search through the study of actual application scenarios, providing some valuable research suggestions for some research projects [15].

## 2. Application and Analysis of Big Data Mining in the Foreign Affairs Translation System

### 2.1. Big Data Mining Technology

Database can provide a lot of information, which brings a lot of benefits to various industries, but it also brings many problems. The most serious problem is that there is too much data, which causes useless information, hides useful information, and does not apply effective knowledge well. Data mining refers to finding valuable rules in massive data and discovering possible laws or relationships. The original database technology can only input, query, and modify the data, cannot find the rules and tendencies, and can lack the ability to mine the hidden information. Data mining technology came into being in this environment.

Data analysis is mainly done by computer. Finding knowledge is to analyze the data, find out the hidden rules, and then use these rules to design the corresponding mining algorithm. Expression and interpretation are realized through various visual forms, such as text, pictures, or tables. Data mining uses artificial intelligence and database technology to extract and analyze complex data and finds valuable information or knowledge through inductive reasoning, so as to help enterprises formulate correct market strategies and reduce decision-making risks. The data and knowledge obtained through excavation can be applied to different industries, such as business management, market production, and engineering design.

#### 2.1.1. Big Data Mining Process

Data mining is unknown, potential, and valuable. It applies the knowledge and experience accumulated by people in the process of processing data to practical problems and turns them into useful information or knowledge. It aims to discover and utilize the hidden knowledge or patterns by analyzing a large amount of meaningful historical data. In enterprise management, it can help managers make correct decisions, so as to increase the quantity of enterprise operation. The data mining model is shown in Figure 1.

Data selection and data set Chengdu should be based on specific operation scenarios. Data mining technology is aimed at specific application background, mining useful information from massive data, which can effectively find out potential patterns and laws and lay the foundation for enterprise decision-making. Data mining stores these information and knowledge into the online transaction processing system or offline data warehouse. In the data selection stage, a large number of bad data are filtered and analyzed to obtain useful data information. These problems can be solved by data cleaning. Data mining is a process of extracting useful knowledge from a large amount of data. Among them, data cleaning plays a vital role in the data analysis ability model.

Data analysis and evaluation are to extract useful information from one or several mining targets, then organize this useful information into a set of data, and finally take this set as the final target result to achieve the desired effect. Data mining is a complex process, which involves many technical problems. Figure 1 shows the statistical process diagram of the data analysis ability model.

### 2.2. Foreign Affairs Translation

There are many countries and nations in the world, and each national has its own specific language and culture. The members of this group carry out dialogue and exchange with each other, which is actually the exchange of various cultures. This kind of cross-cultural communication activity is a social activity that appears only when human society develops to a certain stage. It involves all aspects of politics, economy, culture, and other fields. Foreign affairs translation belongs to the field of cultural exchange. Therefore, foreign affairs translation plays an important role and influence. Foreign affairs translation has a long history, and Bai Guo began to contact foreign affairs translation, which came into being. Foreign affairs translation is to express the meaning of a certain language on a certain foreign affairs discourse in other languages, which conforms to the foreign affairs discourse standard so that the translation can bring the same cognate foreign affairs discourse to the listener and reader as the source language listener or reader.

In today's globalization, foreign affairs activities of exchanges between countries are increasingly frequent. In order to strengthen mutually beneficial cooperation between countries, the advanced experience of other countries should be learnt from and drawn on and the growth of economy and social culture should be increased; it is necessary to interact with people of different languages and cultural backgrounds. With the continuous enhancement of China's economic strength and the rapid improvement of its comprehensive national strength, more and more foreigners began to pay attention to and participated in our foreign affairs. Therefore, it is urgent to strengthen external publicity. Foreign affairs translation is one of the important ways of communication between countries, and it is also an indispensable way for countries to carry out various activities. With the increase of exchanges between countries and the emergence of various forms of cultural exchange, as an important means of communication, foreign affairs translation has gradually become an important cross-cultural communication activity. There is an inseparable relationship between the two.

## 3. Algorithm Formula about Data Search in the Foreign Affairs Translation System

### 3.1. Algorithm Learning of Data Analysis Technology

In the case of massive big data distribution, most data can be gathered in one region, and only a few data are far away. This kind of data is called outlier data. Combined with the characteristics of information technology, the number of users who obtain data through the network is increasing, which leads to data obsolescence. These data usually lead to some wrong conclusions and decisions and even cause serious social problems. Therefore, data mining is needed. Outlier data mining includes text data, spatial data, graph data, and temporal data. When faced with different data types, the appropriate mining methods are also different.

For outlier detection, not all attributes can show data features, and some irrelevant attributes may also be used as main features for detection, which will affect the mining results, resulting in low accuracy of the algorithm. Therefore, different attributes of data are distinguished by weight. The more the weight, the higher the importance. The commonly used weight mathematical formula is as follows:

(1) $$\begin{array}{c} W_{i}=\frac{P_{i}}{\overset{n}{\underset{i=1}{\sum }}P_{i}}\text{,} \end{array}$$

(2) $$\begin{array}{c} W_{i}=\frac{1-E}{k-\sum E_{i}}\text{.} \end{array}$$

In formula (2), *E*_*i*_ represents the information entropy of each attribute, and its value directly affects the influence of different attributes of the data on its weight. The larger the value of *E*_*i*_, the smaller the weight value, indicating that the data attributes occupy less space, that is, the lower the importance. The smaller the value of *E*_*i*_, the larger the weight value, indicating that the data attributes occupy more space, that is, the higher the importance.

In formula (1), *P*_*i*_ represents the number of samples of various properties. When mining outliers, different formulas are given according to the actual application of weight calculation.

The deep forest algorithm (DFA) is one of the algorithms that use forest integration for deep learning. Although this algorithm has made good progress in image processing and other aspects, it has high requirements for training data when training depth models. At the same time, the optimization of a variety of parameters also makes the algorithm very complex. Based on this background, the deep forest algorithm came into being. The node splitting of each subtree under the random forest is achieved by random selection. When the attribute dimension is *m*, the random forest uses the Gini index *g* to represent the node splitting, and the calculation formula is as follows:

(3) $$\begin{array}{c} G=\overset{t}{\underset{i=1}{\sum }}p_{t}\left(1-p_{t}\right)\text{.} \end{array}$$

*p*_*t*_, in formula (3) represents the probability of belonging to class *T* in the data set, which reflects the splitting degree of node splitting index. If the probability of the existence of the *T*-type data set is lower, it indicates that the splitting degree of the node classification index is not high, which indicates that the feasibility of the data set is insufficient, and vice versa.

(4) $$\begin{array}{c} G\left(D,A\right)=\frac{\left|D_{1}\right|}{\left|D\right|}G\left(D_{1}\right)+\frac{\left|D_{2}\right|}{\left|D\right|}G\left(D_{2}\right)\text{.} \end{array}$$

It is any property of data set *D*. According to the original property a, the data set is divided into *D*_1_ and *D*_2_. Each forest generates a *k*-dimensional probability vector and fuses it with the *G*-dimensional original probability vector. The next layer uses the fusion vector as input and uses the *k*-fold cross-validation method to train the data, so as to avoid over-fitting and cross-validation values *β.* The formula is as follows:

(5) $$\begin{array}{c} \beta =\frac{\overset{n}{\underset{i=1}{\sum }}Q_{i}}{n}\text{,} \end{array}$$

where *n* is the number of segmented subsets in the dataset, and *Q*_*i*_ is the result of classification after being segmented by the *i*th one. Finally, the multilayer decision tree algorithm based on the Bayesian network classifier and the hierarchical tree structure is programmed with MATLAB language. The model proposed in this article is simulated and analyzed. The cascade layer iterates in sequence until the maximum number of cascade layers is reached, and the maximum output of the mean value of the probability vector in the forest is taken as the final result.

The idea of filtering the algorithm comes from the combination of things, for example, according to the fact that users have similar hobbies and push the same items to this kind of people.

The algorithm first abstracts the records of the data set as 1 × *N* vectors and then uses the cosine function to calculate the similarity between data sets. The mathematical expression is as follows:

(6) $$\begin{array}{c} sim_{uv}=\cos\;\left(u,v\right)=\frac{u\cdot v}{\left\|u\right\|\left\|v\right\|}=\frac{\underset{i\in uv}{\sum }r_{ui}\times r_{vi}}{\sqrt{\underset{i\in I_{u}}{\sum }r_{ui}^{2}\sqrt{\underset{i\in I_{v}}{\sum }r_{vi}^{2}}}}\text{.} \end{array}$$

In publicity (6), *sim*_*uv*_ represents the calculated value of cosine similarity, which is expressed as the similarity between data sets. The greater the value, the higher the similitude of data sets. On the contrary, the smaller the value, the lower the similitude of the data set, so as to cooperate with the collaborative filtering algorithm to filter the data.

In formula (6), *u* and *V* are the scoring vectors of the data set, ‖*u*‖ and ‖*v*‖ are their vector modulus, *I*_*u*_ and *I*_*v*_ are the similar sets of the data sets *u* and *V,* respectively, and they are the common data sets of the data sets *u* and *V*.

The calculation of cosine similarity is mainly reflected in the inconsistency of vector directions, insensitivity to values, and inconsistency of values in various dimensions of data sets that are difficult to measure. Therefore, the cosine similarity is corrected, and the average score is introduced in the calculation of cosine similarity to reduce the inaccuracy of calculation. The mathematical expression of the modified calculation equation is as follows:

(7) $$\begin{array}{c} sim_{uv}=\frac{u\cdot v}{\left\|u\right\|\left\|v\right\|}=\frac{\underset{i\in I_{uv}}{\sum }\left(r_{ui}-\bar{r_{u}}\right)\times \left(r_{vi}-\bar{r_{v}}\right)}{\sqrt{\underset{i\in I_{u}}{\sum }{\left(r_{ui}-\bar{r_{u}}\right)}^{2}}\sqrt{\underset{i\in I_{v}}{\sum }{\left(r_{ui}-\bar{r_{v}}\right)}^{2}}}\text{.} \end{array}$$

### 3.2. Analysis of the K-Means Clustering Algorithm

Cluster analysis, as a theory of studying and analyzing data structure, has been accepted and widely used in the field of pattern recognition and data processing. Cluster analysis has been paid more and more attention and widely used in various fields.

The K-means algorithm is one of the most simple and universal representative algorithms in hard clustering algorithms. It first selects the initial cluster center, then calculates the distance from the remaining samples to each cluster center, and classifies the samples into the category of the nearest cluster center. The average value of each class or cluster should be recalculated according to formula (8) until the criterion function tends to be consistent.

(8) $$\begin{array}{c} c_{j}=\frac{1}{n_{j}}\overset{n_{j}}{\underset{i=1}{\sum }}x_{i}\text{,} \end{array}$$

(9) $$\begin{array}{c} E={\overset{k}{\underset{i=1}{\sum }}\underset{x\in C_{i}}{\sum }\left|x-\bar{x_{i}}\right|}^{2}\text{.} \end{array}$$

### 3.3. Analysis of the Fuzzy c-Means Clustering Algorithm

In order to mark that sample *kx*_*k*_ belongs to class I, this article defines *u*_*ik*_ and satisfies condition 0 ≤ *u*_*ik*_ ≤ 1. Therefore, *b* = 1/2. In this article, we apply fuzzy set theory to the study of clustering problems. This method is proved to be effective by clustering an actual data set. It is general and practical. The objective function is defined as follows:

(10) $$\begin{array}{c} J\left(U,V\right)=\overset{n}{\underset{k=1}{\sum }}\overset{c}{\underset{i=1}{\sum }}u_{ik}^{m}d_{ik}^{2}\text{.} \end{array}$$

In formula (10), *U*=(*u*_*ik*_)_*c∗n*_ is the auxiliary matrix, *d*_*ik*_=‖*x*_*k*_ − *v*_*i*_‖. *J*(*U*, *V*) represents the M-power of the degree of attachment from the data set to the computing center, and the process is as follows:

(1) We calculate the clustering center *V* in step 1 by using the following formula:
  (11) $$\begin{array}{c} v_{i}=\frac{\overset{n}{\underset{k=1}{\sum }}{\left(u_{ik}^{\left(l-1\right)}\right)}^{m}x_{k}}{\overset{n}{\underset{k=1}{\sum }}{\left(u_{ik}^{\left(l-1\right)}\right)}^{m}}\text{.} \end{array}$$
(2) We correct the subordinate matrix *U* and calculate the objective function *J*; its mathematical expression is as follows:
  (12) $$\begin{array}{c} U_{ik}={\left[\overset{\varepsilon }{\underset{j=1}{\sum }}{\left(d_{ik}/d_{jk}\right)}^{\frac{2}{m-1}}\right]}^{-1}\text{,}\\ J\left(U,V\right)=\overset{m}{\underset{k=1}{\sum }}\overset{c}{\underset{i=1}{\sum }}{\left(u_{ik}\right)}^{m}{\left(d_{ik}\right)}^{2}. \end{array}$$

Through the above formula calculation, the clustering center *V*, the auxiliary matrix *U*, and the minimum objective function value can be obtained. When *u*_*jk*_=max_1≤*c*≤*i*_{*u*_*ik*_}, sample *x*_*k*_ can be classified as *J*.

### 3.4. Analysis of the BP Neural Network Algorithm

BP process determines the weight of the connection between nodes on the basis of data training and calculates the minimum mean square error (MMSE) between the actual value and the estimated value from the output. Its purpose is to minimize the total error (i.e., the average error) of the network calculation output. On this basis, the artificial neural network is applied to short-term load forecasting. The improved genetic algorithm is used to optimize the weight. Combined with the BP algorithm, the adaptive learning of the BP model is realized.

Suppose the neural network contains *D* neurons in the input layer, *Q* neurons in the hidden layer, and *l* neurons in the output layer. On this basis, a radial basis function neural network model with three-layer structure is established. Simulation experiment displays that the system could effectively deal with the problem of edge extraction under noise interference, and the training speed is fast and easy to realize. In view of the slow convergence speed and easy to fall into local minima of the BP network, an improved genetic algorithm (GA)-based optimized RBF neural network is proposed for image edge detection. The input of the input layer to the *H* neuron of the hidden layer is indicated as follows:

(13) $$\begin{array}{c} a_{h}=\overset{d}{\underset{i=1}{\sum }}v_{ih}x_{i}\text{.} \end{array}$$

Then, mark on the *j*th neuron input from the hidden layer to the output layer as follows:

(14) $$\begin{array}{c} \beta_{j}=\overset{d}{\underset{i=1}{\sum }}w_{jh}b_{n}\text{.} \end{array}$$

*β*_*j*_ is the output result marking of the *j*th neuron of the output layer by the hidden layer. The marking result is that the neuron in the neural network accepts the input from other neurons and multiplies these by the corresponding weight. The marking index of the output result can compare and analyze the total input and the threshold to judge the weight relationship between the data nodes.

Ideally, the activation function should be a step function, but the step function has problems such as discontinuity, nondifferentiability, and nonsmooth points, so it is usually replaced by sigmoid function, and its mathematical expression is as follows:

(15) $$\begin{array}{c} sgn\left(x\right)=\left\{\begin{array}{cc} 1\text{,} & x\geq 0\text{,}\\ 0\text{,} & x\leq 0\text{,} \end{array}\right.\\ \mathrm{sigmoid}\left(x\right)=\frac{1}{1+e^{-x}}\text{.} \end{array}$$

For neural network training sample (*x*_*k*_, *y*_*k*_), we assume that the output variable is Y, and its output expression is represented by equation (16), where *f* is the sigmoid activation function, and (*x*_*k*_, *y*_*k*_) calculates the representation of the mean square error in the network (17).

(16) $$\begin{array}{c} Y_{j}^{k}=f\left(\beta_{j}-\theta_{j}\right)\text{,} \end{array}$$

(17) $$\begin{array}{c} E_{k}=\frac{1}{2}\overset{n}{\underset{j=1}{\sum }}{\left(Y_{j}^{k}-y_{j}^{k}\right)}^{2}\text{.} \end{array}$$

In the case of random given parameter set, the BP algorithm is used to continuously update the parameters until the appropriate set value *E*_*k*_ is obtained, so that *E*_*k*_ takes the extreme value, and then the neural network training ends. This method is applied to nonlinear system identification and compared with the least square method and the recursive formula method.

## 4. Experimental Analysis of the Application of Data Search in the Foreign Affairs Translation System

### 4.1. Experimental Analysis of Big Data Mining Algorithm Technology

By using FIMI repository accidents, Kosarak, and Webdocs, the dataset gets Table 1.

As shown in Table 1, the characteristic statistics of the data sets are shown, and the specific attributes of the three data sets are counted from four aspects as follows: average length, number of items, number of transactions, and size.

#### 4.1.1. Comparison of Running Time of the Big Data Mining Algorithm

The runtime performance of PrePost, Fidoop, and growth is compared and analyzed. In addition, this article also tests three test data sets and multiple minimum support thresholds.

As shown in Figure 2, compared with Fidoop, Fidoop uses FIU tree structure to mine frequent itemsets, generates all possible *K* itemsets by solving each transaction record, and constructs *K* itemsets with the same length as a k-fitree structure, so as to avoid the time overhead required by recursively constructing and traversing massive conditional FP trees, and the algorithm performance is generally faster than growth. A distributed data mining method based on support vector machine classification is proposed.

As shown in Figure 3, compared with PFP growth, Mrprune PrePost reduces the loss of time problem caused by forming many frame containers and constructing a large number of conditional FP trees on the basis of n-list cross operation. The cross-operation efficiency in *n*-list is very high.

Figure 4 displays the statistical figure of running time on Webdocs data group. It can be seen from the data in the chart that the running time of the three data sets increases with the decline of the minimum support rate.

Figures 2to 4 show that for each data set and each minimum support threshold, PrePost is the fastest algorithm among all algorithms. For high minimum support threshold, Fidoop usually runs faster than growth. For low minimum support threshold, Fidoop is more time-consuming. For low minimum support threshold, PrePost has more obvious advantages.

#### 4.1.2. Comparison of Memory Consumption of the Big Data Mining System

As shown in Figure 5, for all data sets, among various algorithms, growth consumes the least memory, followed by PrePost, but there is little difference between the two. By comparing and discussing the experimental results, we found that under the same conditions, it has better performance than the other two methods. Even though the memory consumption of PrePost is greater than that of growth, as analyzed in the runtime experiment, its consumption of runtime is less than that of growth.

Compared with growth, the nodes of PPC tree in the tree structure of PrePost contain other additional information, resulting in PPC tree constructed from the same dataset occupying more memory than pf tree constructed. In addition, PrePost finds frequent itemsets based on n-list, which is composed of a series of PP codes, which will also increase additional memory consumption.

### 4.2. Experimental Analysis on the Application of Big Data Mining Technology in the Foreign Affairs Translation System

For better inspection function of the foreign affairs translation system, on the test of a large number of translation data, this article takes small document text data as the main processing object, processing a total of 22573 small documents, and the data size ranges from a few KB to a few MB.

As shown in Figure 6, the running time of the number of translated texts for different foreign affairs fluctuates. The translation time of the number of texts from the range of [10–20] KB to the range of [90–100] KB shows a downward trend. After the number of texts is greater than 100 kb, the translation time of texts between 90 and 100 kb increases significantly.

The default data blocks of all files are small files, and the amount of data in a few kilobytes is very small, which also reduces the proportion of tasks that only consume system resources and almost does not process data in the overall time consumption. 10–100 kb occupies most of the data of the test data, which tests the accuracy of the small file processing means in this article. Text data volume greater than 100 kb also accounts for a part of the total data. The data simulates the real patent data volume.

In order to test the accuracy of the experiment, the traditional, NS, and optimized ns methods are compared and analyzed, and the time efficiency is compared. On this basis, the improved Morse Chang method is used for numerical simulation. From the simulation analysis, it can be seen that the new method proposed in this article has high speed and accuracy and is easy to implement with less calculation.

As shown in Table 2, the processing method using MapReduce can significantly improve the translation processing efficiency, which is about 5.8 times that of the traditional method. The reason is that MapReduce can use the characteristics of clusters to realize the purpose on parallel processing, and the method used in this article is better than MapReduce, which can improve the translation efficiency by about 5 times, because the method in this article will reduce the occupation of system allocation resources when translating patent data.

As shown in Figure 7, to test the feasibility of the method in dealing with small files compared with other small files, the archived file method and the serialized file method are studied and compared. In terms of test settings, the size of the block is set to 50 kb. The results show that under the same conditions, the two methods have no significant difference in data size, arrangement order, and storage space. However, in terms of computational efficiency, the former is higher than the latter. Therefore, the filing method has more advantages in application. The size of each combined fragment of this research method is 200 KB, and the serialized file can be segmented. The experimental results are shown in Table 3.

As shown in Table 3, the data show that when different kinds of data translate text files and file sizes are different, the text translation processing time rises with the raise of the quantity and size of files. Each type of translated text file leads to a different increase in translation processing time, among which the increase of this method is the highest and that of archived files is the lowest.

It can be seen that serialized files have better processing effect, and scattered files can be processed in a centralized manner to reduce the number of small files. This method has the best effect in processing time, but the most obvious disadvantage of this method is that it cannot reduce the memory of small files in the management node.

As shown in Figure 8, the processing time of archive file is not much different from that of the NS mode. Even though the processing efficiency is still low, the reason is that the archive file method is a secondary index structure, which will spend some time reading files. The advantage of this method is that it can reduce the memory of the management node.

As shown in Table 4, based on the increase of text size, the quantity of maps increases exponentially with time. This test fully proves that the speed of data translation processing performance is closely related to file size under the influence of file size parameters.

As shown in Figure 9, it is not shown that more amount of fragmented data are merged, which has a certain relationship with the processing speed of the translation engine. When the amount of fragmented data is large, the corresponding parallelism is small. At this time, it is necessary to weigh the allocation of map time and parallelism. Blindly increasing the amount of fragmented data cannot achieve the best result. From the test in the text, the best result can be achieved when the amount of fragmented data is 100 kb.

## 5. Conclusion

First, it introduces the growth of data analysis ability and overview of big data mining theory, as well as the process of big data mining and introduces the meaning and importance of the foreign affairs translation system. Then, it puts forward the research background of the project and direction of this topic, focusing on the application analysis of the foreign affairs translation system based on big data analysis ability. Then, it introduces the algorithm formula based on big data mining in the foreign affairs translation system, mainly including the data analysis ability algorithm, K-means clustering formula analysis, fuzzy average interaction, and neural network formula analysis. Finally, the application of data analysis ability in foreign affairs translation system is investigated and analyzed. It is verified that the combination of big data mining technology and foreign affairs translation system application can better promote the universality, efficiency, and high fault tolerance of the foreign affairs translation system, and the experimental investigation results are sorted out and classified.

## Figures and Tables

**Figure 1:** Process diagram of the data analysis ability model.

**Figure 2:** Running time statistics on data set accidents.

**Figure 3:** Running time on Kosarak dataset.

**Figure 4:** Running time on Webdocs dataset.

**Figure 5:** Memory consumption on three data sets.

**Figure 6:** Statistics on the number of translated texts of foreign affairs.

**Figure 7:** Comparison of translation processing methods.

**Figure 8:** Comparison of translation processing methods.

**Figure 9:** Relationship between translation time and number of slices.

**Table 1:** Similarity analysis between data groups.

Data groups	Average length	Number of projects	Number of transactions	Size
Accidents	33.8	468	240183	35.5
Kosarak	8.1	41270	990002	32.1
Webdocs	40.5	526765	169208	1515.5

**Table 2:** Data translation processing performance test I.

File size	Processing time (s)	Mr processing method		Paper method	
		Number of maps	Time/s	Number of maps	Time/s
100 KB	198	10	45	1	290
1 MB	2593	30	453	5	488
10 MB	25688	293	4451	45	3662
20 MB	51576	534	8665	112	7324
40 MB	104263	916	18621	216	14732

**Table 3:** Data translation processing performance test II.

File size	Archive documents		Serialize file		Paper method	
	Number of maps	Time/s	Number of maps	Time/s	Number of maps	Time/s
10 KB	1	29	1	30	1	36
100 KB	10	46	2	152	1	291
1 MB	30	464	20	469	5	485
10 MB	293	4462	200	3953	45	3672

**Table 4:** Data translation processing performance test III.

File size	50 KB		100 KB		200 KB		400 KB		800 KB	
	Quantity	Second	Quantity	Second	Quantity	Second	Quantity	Second	Quantity	Second
20 KB	1	49	1	49	1	45	1	49	1	43
200 KB	4	132	2	310	1	517	1	516	1	519
2 MB	40	630	20	600	10	669	5	727	3	906
20 MB	400	6345	200	6132	100	6553	50	7053	25	7863

## Data Availability

The experimental data used to support the findings of this article are available from the author upon request.
